The article "Application Effect of Sevoflurane Combined with Nerve Block Anesthesia in Surgical Anesthesia in Patients with Uterine Fibroids" was published in 2022. Journal: Contrast Media Mol Imaging.

# Application Effect of Sevoflurane Combined with Nerve Block Anesthesia in Surgical Anesthesia in Patients with Uterine Fibroids

**DOI:** 10.1155/2022/9983851

**Published:** 2022-06-24

**Authors:** Shujing Fan, Shiduo Li

**Affiliations:** ^1^Obstetrics and Gynecology, Yan'an People's Hospital, Yan'an, Shaanxi 71600, China; ^2^Anesthesiology Department, Yan'an People's Hospital, Yan'an, Shaanxi 71600, China

## Abstract

Sevoflurane has been widely used clinically as an inhalation anesthetic. A review of domestic and domestic research, combined with the current synthesis research, pharmacological progress, existing production capacity, production, and sales status, can show that sevoflurane is a very good new type of inhalation anesthetic. *Objective*. To study the effect of sevoflurane combined with nerve block anesthesia on stress response and hemodynamics in patients with uterine fibroids surgery. *Methods*. We selected 100 cases of myomectomy patients as the research objects and divided them into observation and control groups according to the random number table method, with 50 cases in each group. The comparison group received propofol combined with remifentanil intravenous compound anesthesia, while the observation group received sevoflurane combined with nerve block anesthesia. The stress response and hemodynamic changes were compared between the two groups 5 minutes before anesthesia (T1), 30 minutes after pneumoperitoneum (T2), and at the end of the operation (T3). At the same time, the differences in cognitive function and adverse reactions were also compared 1 day before surgery and 1 day after surgery. *Results*. At T2 and T3, the stress response indexes of cortisol, epinephrine, norepinephrine, and blood sugar in the observation group were lower than those in the control group. In addition, hemodynamic indicators heart rate, mean arterial pressure, and blood sample saturation levels were also lower than those in the control group. One day after the operation, the score of the Simple Mental State Scale in the observation group was higher than that in the control group, and the time phrase for the completion of the connection test was in the control group. The incidence of adverse reactions in the observation group was lower than that in the comparison group. *Conclusion*. Sevoflurane combined with nerve block anesthesia in patients undergoing myomectomy can significantly reduce the body's response to hormones, maintain hemodynamic stability, reduce cognitive impairment, and help avoid adverse reactions.

## 1. Introduction

In recent years, it has been found that fluorinated ethers have effective inhalation anesthesia. Included among these anesthetics are desflurane (CF3CHFOCHF3), isoflurane (CF3CHCIOCHF2), enflurane (C1FCHCH2OCHF2), and sevoflurane (CF3CHOCH2F) [1]. Due to its rapid loss of consciousness and rapid recovery, sevoflurane is a desirable property of contemporary inhalation anesthetics, making it a particularly advantageous inhalation anesthetic. About 1% to 5% by volume of a mixture with oxygen or a gaseous mixture containing sufficient oxygen to maintain the respiratory volume is provided by the inhalation route to air-breathing mixed-breed animals. Inhalation anesthetics [2–4] have the following advantages. First, the concentration of anesthetics in the blood (or called partial pressure) can be effectively adjusted by breathing, and in particular, the inhaled anesthetics can be quickly washed out of the body. Second, the concentration (partial pressure) of the inhalation anesthetic at its site of action (central nervous system) can be estimated by measuring the end-tidal concentration. It is precisely because of these two advantages that inhalation anesthesia has received more and more attention in general anesthesia for surgery. Subsequently, the demand for sevoflurane has gradually increased. Sevoflurane has been included in the scope of national medical insurance, so the market demand for sevoflurane is wide, and the prospect is huge.

The article "Application Effect of Sevoflurane Combined with Nerve Block Anesthesia in Surgical Anesthesia in Patients with Uterine Fibroids" was published in 2022. Journal: Contrast Media Mol Imaging.

Sevoflurane is a new type of inhalation anesthetic with few side effects and a broad market prospect. According to statistics, the total global sales of sevoflurane in 2003 reached 500 million US dollars. Due to its mask-induced convenience and reliable cardiovascular safety, it has been widely used abroad. China has long relied on importing sevoflurane from abroad for clinical use. Many experiments have shown that sevoflurane has a very low blood gas partition coefficient (only a few percent of that of halothane and isoflurane), rapid induction, and stable hemodynamics. Its respiratory depressant and cardiovascular system effects are smaller than isoflurane. Other than that, sevoflurane does not cause allergic reactions and is mildly irritating to the mucous membranes of the eyes. The depth of anesthesia of sevoflurane can be easily adjusted, which is an ideal characteristic of contemporary inhalation anesthetics and is a very good new type of inhalation anesthetics [4].

Uterine fibroids [5, 6] are mostly manifested as abdominal pain, heavy menstrual flow, and even anemia that requires blood transfusion. Surgery remains the preferred treatment option for patients with severe uterine fibroids. However, surgical stress can significantly affect the patient's physiological and information status, which is not conducive to postoperative recovery [7]. The perioperative stress response is mainly caused by surgical trauma and anesthesia. Changes in sympathetic excitability and cortisol concentrations can lead to increased blood pressure and increased heart rate, increasing the risk of anesthesia and surgery. In addition to causing a certain degree of stress to the patient, surgery also causes hemodynamic disturbances in the body, which in turn threatens the patient's life and health [8]. Laparoscopic surgery, as one of the most common minimally invasive surgical methods, has the advantages of less trauma, less pain, and quicker postoperative recovery and has been widely used in gynecological surgery [9]. However, laparoscopic surgery can still cause a certain stress response, which will significantly affect the patient's respiratory and circulatory systems, and even affect their hemodynamics and cognitive function [10]. Therefore, seeking a safe and efficient operation and anesthesia is particularly important for patients with uterine fibroids. As an inhalation general anesthetic, sevoflurane has significant advantages in induction speed, anesthesia efficacy, and blood gas partition coefficient. Nerve block anesthesia is a commonly used anesthesia induction and maintenance agent in clinical surgery, with strong analgesic effect, short half-life, and less impact on cardiovascular [11]. Some researchers have found that the combined application of these two methods during anesthesia can effectively reduce adverse stress reactions during surgery, but there are few studies on their combined application. Therefore, this study used sevoflurane combined with nerve block anesthesia to observe its effects on stress response and hemodynamics in patients undergoing myomectomy.

The article "Application Effect of Sevoflurane Combined with Nerve Block Anesthesia in Surgical Anesthesia in Patients with Uterine Fibroids" was published in 2022. Journal: Contrast Media Mol Imaging.

## 2. The Review of Research Progress

### 2.1. Source and Production and Sales Status

Sevoflurane was synthesized by Regan in 1968 and was first reported by Willin et al. in 1971. The physicochemical properties, pharmacological effects, and toxicology were evaluated in 1975 [12]. In the 1960s, sevoflurane was researched and synthesized by Baxter Pharmaceuticals in the United States. Abbott Corporation officially listed it in June 1995. At present, the production capacity of domestic production enterprises in anesthetics is relatively limited, mainly including ketamine, sodium oxybate, anesthetic ether, and midazolam. In 1998, the total sales volume was less than 250 million CNY. Among these drugs, only anesthetic ether is an inhalation anesthetic. In 1998, in the world's top 100 prescription drugs, the combined sales of the two general anesthetics reached 1.17 billion US dollars.

At present, the inhalation anesthetics listed in China mainly include nitrous oxide, chloroalkane, anesthetic ether, and isochlor ether. China has been relying on imported sevoflurane from abroad for clinical needs. Experiments show that sevoflurane has a very low blood gas partition coefficient and is hemodynamically stable. Due to its good anesthetic properties and small side effects, sevoflurane has quickly become a substitute for many anesthetics and has a very broad market prospect. In China, Jiangsu Hengrui obtained the approval number of SFDA in June 2004. Lunan Pharmaceutical Group Co., Ltd. obtained the approval number in 2008.

The article "Application Effect of Sevoflurane Combined with Nerve Block Anesthesia in Surgical Anesthesia in Patients with Uterine Fibroids" was published in 2022. Journal: Contrast Media Mol Imaging.

### 2.2. Pharmacological Research Progress

Clinically, sevoflurane is used as a general anesthetic. During induction of anesthesia, 50%∼70% nitrous oxide and 2.5%∼4% of this product are inhaled. Intravenous anesthesia with sleeping doses is usually induced at 0.5% to 5%. When used as anesthesia maintenance, surgical anesthesia should be maintained at the lowest effective concentration, usually below 4%. Sevoflurane is an anesthetic that has entered the clinic in recent years with rapid induction, no odor, and easy-to-control anesthesia depth. After two minutes of induction with 4% sevoflurane and oxygen mask inhalation, the patient will lose consciousness. At the same time, rhythmic slow waves will appear in the patient's brain waves. With the deepening of anesthesia, the slow waves gradually decrease, and a spike-like wave group appears similar to that of barbiturates. Sevoflurane inhibits the reticular neurons of the midbrain in a concentration-dependent manner. Deep anesthesia may cause systemic spasm, but no obvious spasticity has been found clinically. Sevoflurane is not irritating to the respiratory tract and does not increase respiratory secretions. With the deepening of anesthesia, sevoflurane can increase respiratory depression, reduce tidal volume, decrease functional residual capacity, increase respiratory rate, and increase PaCO2 [13, 14]. In terms of liver function effects, sevoflurane produces less liver damage and has a stronger muscle relaxation effect. The low solubility of sevoflurane in blood results in a rapid rise in alveolar drug concentrations during induction of anesthesia and a rapid decline after cessation of inhalation. Less than 5% of sevoflurane in humans is absorbed and metabolized. Rapid and extensive pulmonary clearance of sevoflurane reduces its metabolizable amount. Transient increases in plasma inorganic fluoride levels occur during and after sevoflurane anesthesia. Typically, inorganic fluoride concentrations peak within 2 hours after sevoflurane anesthesia and return to preoperative levels after 48 hours. The blood concentration of sevoflurane reaches a steady state 10–15 minutes after inhalation and disappears after inhalation. It is mainly excreted through exhalation, and about 40% of the original drug is excreted in exhalation 1 hour after inhalation is stopped, and the disappearance rate in the body is greater than that of enflurane. Sevoflurane can significantly enhance the muscle relaxant effect of nondepolarizing muscle relaxants. Therefore, when using sevoflurane, the dose of these drugs should be adjusted appropriately. Similar to isoflurane, sevoflurane requires the addition of epinephrine when exogenous arrhythmias occur due to myocardial sensitization. Similar to other drugs, sevoflurane can reduce its concentration when combined with intravenous anesthetics such as propofol. CYP2E1 inducers increase the metabolism of sevoflurane but not barbiturates [15].

The article "Application Effect of Sevoflurane Combined with Nerve Block Anesthesia in Surgical Anesthesia in Patients with Uterine Fibroids" was published in 2022. Journal: Contrast Media Mol Imaging.

## 3. Materials and Methods

### 3.1. Normal Information

In this paper, we selected 100 patients who were scheduled to undergo laparoscopic myomectomy in Zhongda Hospital Affiliated to Southeast University in Pukou District, Nanjing, from August 2019 to December 2020 as the research subjects. All cases were divided into observation group and control group by random number table method, 50 cases in each group. The age of the observation group was 36–60 years old, with an average of 42.32 ± 5.01; the weight was 51–69 kg, with an average of 58.73 ± 5.21 kg. The course of disease was 16–24 months, with an average of 19.05 ± 0.87 months. The fibroids were 3–8 cm in size, with an average of 5.04 ± 0.79 cm. The age of the control group was 37–61 years old, with an average of 42.35 ± 5.02; the weight was 52–70 kg, with an average of 58.76 ± 5.25 kg. The course of disease was 17–25 months, with an average of 19.08 ± 0.89 months. The fibroids were 4–8 cm in size, with an average of 5.05 ± 0.80 cm. There were statistically significant differences in general clinical resources such as age, weight, course of disease, and size of fibroids between the two groups (*P* > 0.05), which were comparable. All patients in this study gave informed consent and were approved by the Ethics Committee of Zhongda Hospital Affiliated to Southeast University, Pukou District, Nanjing City. In detail, the comparison of the general clinical data of the two groups of patients is shown in Table 1.

### 3.2. Standard Constraints

Inclusion criteria are as follows: ① clinically diagnosed with uterine fibroids, in line with surgical indications; ② no neurological or serious cardiovascular disease; ③ normal coagulation function; ④ patients with American Society of Anesthesiologists (ASA) grades I-II; ⑤ body mass index <30 kg/m^2^; ⑥ voluntarily participating in this study and signing the informed consent. This study was approved by the hospital's ethics committee.

The article "Application Effect of Sevoflurane Combined with Nerve Block Anesthesia in Surgical Anesthesia in Patients with Uterine Fibroids" was published in 2022. Journal: Contrast Media Mol Imaging.

Exclusion criteria are as follows: ① severe peptic ulcer bleeding; ② severe liver and kidney dysfunction; ③ respiratory and circulatory system diseases; ④ patients with diabetes and immune system diseases; ⑥ preoperative and intraoperative blood transfusion; ⑦ abdominal surgery history; ⑧ suffering from other tumors; ⑨ preoperative cognitive dysfunction or mental disorder.

### 3.3. Method

The patients in both groups were routinely fasted for 12 hours before operation; water was forbidden for four hours before operation, and they were not given any drugs. After entering the operating room, the right upper extremity venous access was established, and 10–15 ml (kg.h) of lactated Ringer's solution was infused. The heart rate, mean arterial pressure, blood oxygen saturation, systolic blood pressure, electrocardiogram, and bispectral index of EEG were monitored by multifunctional monitor. All patients received oxygen inhalation at 2.5 L/min through a mask and underwent general anesthesia. Vecuronium bromide 0.1 mg/kg, midazolam 0.05 mg/kg, and remifentanil 2–3 *μ*g (kg h) were intravenously injected sequentially. The drugs used for injection in this study were all produced by Jiangsu Enhua Pharmaceutical Co., Ltd. Its production batch number is 20170630, and the specification is 1 mg. The target control concentration of remifentanil was set to 3 ng/ml, and the induction was maintained for 2–3 minutes. After muscle relaxation, tracheal intubation was performed, and mechanical ventilation was performed in parallel. The tidal volume was 8–12 mL/kg, the oxygen flow was 2.5 L/min, and the respiratory rate was 10–14 times/min. At the same time, we controlled the pneumoperitoneum pressure at 12∼14 mmHg. During the maintenance of anesthesia, the control group received intravenous injection of propofol 4–8 mg/(kg.h), and the observation group was in line with the inhalation of 1.5%–3.0% sevoflurane. The sevoflurane was produced by Shanghai Hengrui Pharmaceutical Co., Ltd., the production batch number was 20170823, and the specification was 120 mL. Both groups were given intermittent injection of rocuronium bromide 5–10 mg/time to maintain the muscle relaxation effect. The BIS value was maintained at 40∼60. We adjusted the drug concentration in a timely manner according to the intraoperative needs to maintain the optimal depth of anesthesia. Anesthetics were discontinued after the operation, and the patient recovered spontaneous breathing and consciousness and was extubated. Circulating blood pressure in both groups was maintained in the range of 90–140/60–90 mmHg, and vasoactive drugs were not used to control blood pressure. Local injection of 2% lidocaine hydrochloride 3∼5 mL relieves incision pain. For patients with HR deceleration <50 beats/min or blood pressure, we decreased ≥20% during surgery, and the concentration of remifentanil and sevoflurane should be reduced. If severe nausea, vomiting, and irritability occur after surgery, the symptoms are relieved by injection of compound aminolimbarbital, and flurbiloride 50 mg intravenously is given for analgesia.

The article "Application Effect of Sevoflurane Combined with Nerve Block Anesthesia in Surgical Anesthesia in Patients with Uterine Fibroids" was published in 2022. Journal: Contrast Media Mol Imaging.

### 3.4. Observation Indicator

The stress response and hemodynamic changes were compared between the two groups at five minutes before anesthesia (T1), 30 minutes after pneumoperitoneum (T2), and at the end of the operation (T3). Differences in cognitive function and adverse reactions 1 day before surgery and 1 day after surgery also need to be compared. The stress response was mainly assessed by detecting the levels of cortisol (COR), epinephrine (A), norepinephrine (NA), and blood glucose (GLU). The levels of COR, A, and NA were detected by radioimmunoassay, and the kits were purchased from Shanghai Hengyuan Biotechnology Co., Ltd. GLU levels were detected by a Roche ACCU-CHEK blood glucose meter. Hemodynamic changes were mainly assessed by measuring heart rate (HR), mean arterial pressure (MAP), and blood oxygen saturation (SpO2) levels. Among them, HR and MAP were detected by the Hungarian Linear Technology LABTECH Kft electronic recorder, and SpO2 was detected by the American OPTI blood gas analyzer. Cognitive function was assessed using the Mini-Mental State Inventory (MMSE) and the Wiring Test (TMT). Among them, MMSE mainly includes language comprehension ability, memory function, computing ability, and time orientation. The total score is 30 points, and the higher the score, the better the cognitive function of the patient [16]. TMT mainly refers to distributing the numbers 1–25 on a white paper and recording the time it takes for the patient to connect the numbers in order from small to large. The shorter the time, the better the cognitive function of the patient. Adverse reactions were assessed by dizziness, nausea and vomiting, and agitation.

### 3.5. Statistical Processing

We used chi-square test, *t*-test, analysis of variance, and SNK test to analyze the data.

We used SPSS 21.0 software for statistical analysis. Measurement data were expressed as mean ± standard deviation, which was in line with the homogeneity of variance. The *t*-test was used for comparison between groups, and the repeated measures analysis of variance was used for comparison at different time points. Further pairwise comparisons were performed using the SNK test. Enumeration data were expressed as rate (%), and chi-square test was used for comparison between groups. *P* < 0.05 was considered significant difference.

The article "Application Effect of Sevoflurane Combined with Nerve Block Anesthesia in Surgical Anesthesia in Patients with Uterine Fibroids" was published in 2022. Journal: Contrast Media Mol Imaging.

## 4. Experimental Results and Analysis

### 4.1. Result Analysis

There was no significant difference in anesthesia induction time, operation time and intraoperative blood loss between the two groups. The detailed results are shown in Table 2.

#### 4.1.1. Comparison of Two Groups of Stress Response Indicators

At T1 time point, there was no significant difference in serum COR, A, NA, and GLU levels between the two groups (*P* > 0.05). At T2 and T3 time points, the levels of COR, A, and NA in the two groups were significantly increased, and the difference was significant (*P* < 0.05). The levels of COR, A, NA, and GLU in the observation group at T2 and T3 time points were significantly lower than those in the control group (*P* < 0.05). The detailed experimental comparison results are shown in Table 3.

#### 4.1.2. Comparison of Hemodynamic Indexes between Two Groups

At T1 time point, there was no significant difference in HR, MAP, SPO2, and other hemodynamic indexes between the two groups (*P* > 0.05). At T2 and T3 time points, HR and MAP in the two groups were significantly increased, and the difference was significant (*P* < 0.05). HR, MAP, and SPO2 in the observation group at T2 and T3 time points were significantly lower than those in the control group, and the difference was significant (*P* < 0.05). The detailed comparison results are shown in Table 4.

#### 4.1.3. Comparison of Cognitive Function between Two Groups

There was no significant difference in cognitive function between the two groups one day before surgery (*P* > 0.05). One day after the operation, the MMSE score of the observation group was significantly higher than that of the control group, and the completion time of TMT was significantly shorter than that of the control group, and the difference was significant (*P* < 0.05). The detailed comparison results are shown in Table 5.

#### 4.1.4. Comparison of Adverse Reactions between the Two Groups (N = 50)

The incidence of adverse reactions in the observation group (8.33%) was significantly lower than that in the control group (21.67%), and the difference was significant (*P* < 0.05). The detailed comparison results are shown in Table 6.

### 4.2. Discussion

Laparoscopic myomectomy is an effective method widely used in clinical treatment of uterine fibroids, with the characteristics of less trauma, fewer postoperative complications, and faster postoperative recovery. However, it is still one of the invasive treatment methods, which will cause different degrees of stress response to the patient and may cause hemodynamic disturbances. It is particularly important to choose a reasonable and effective anesthesia method, and it is also the key to ensure the successful completion of the operation. Remifentanil is a new type of anesthetic that is widely used in clinical practice. It has the advantages of rapid onset of action and rapid clearance. Relevant research reports show that remifentanil has a short half-life and will not accumulate in the body, which is beneficial to shorten the patient's breathing recovery time and will not affect the patient's quality of recovery. In the past, propofol and remifentanil anesthesia were mainly used in clinical anesthesia for patients undergoing laparoscopic hysterectomy. Although this anesthesia program can achieve relatively obvious effects, it has a great impact on the cognitive function of patients, and is likely to cause a series of adverse reactions such as coma, dizziness, vomiting, and drowsiness. Therefore, this anesthesia protocol has significant limitations. Some clinical studies believe that propofol has a strong cardiovascular inhibitory effect when used for anesthesia and sedation maintenance. For patients with preexisting hypertension and heart disease, it may lead to intraoperative hypotension and circulatory instability. Because most of the anesthesia in laparoscopic myomectomy is simple general anesthesia, lack of adequate analgesia can easily cause hemodynamic changes. The blood concentration of fentanyl used in the past is unstable, and repeated additions are likely to cause accumulation. When the BIS is controlled within 60, sufficient analgesic effects cannot be ensured.

The article "Application Effect of Sevoflurane Combined with Nerve Block Anesthesia in Surgical Anesthesia in Patients with Uterine Fibroids" was published in 2022. Journal: Contrast Media Mol Imaging.

Sevoflurane is one of the new types of inhalation anesthetics. It has the characteristics of stable MAC value, fast onset, rapid elimination, no obvious inhibition of cerebrovascular autoregulation, good cardiovascular stability, and less respiratory irritation. Its blood volatility and solubility are low, and its application in clinical anesthesia is remarkable. Previous animal studies have shown that sevoflurane has a protective effect on the hypoxic stress process of cardiac cells and nerve cells. Its main principle of action may be to protect the function of cells by scavenging the generation of oxygen free radicals under hypoxia. Studies have shown that when sevoflurane is used for anesthesia in patients with cerebral hemorrhage, their circulating blood pressure is more stable, and the secretion of oxidative stress substances such as superoxide dismutase in serum is significantly lower than that in the traditional intravenous anesthesia group. Since sevoflurane and propofol have different anesthesia methods, there is some controversy about their anesthesia effects in clinical practice. Therefore, this study observed the effects of propofol and sevoflurane combined nerve block anesthesia on stress response and hemodynamics in patients. Through these studies, the clinical strategies to improve the intraoperative anesthesia effect and surgical safety of patients with uterine fibroids were explored.

The article "Application Effect of Sevoflurane Combined with Nerve Block Anesthesia in Surgical Anesthesia in Patients with Uterine Fibroids" was published in 2022. Journal: Contrast Media Mol Imaging.

The results of this study showed that there was a certain degree of stress response in both groups during the operation, and the hemodynamics also changed to varying degrees. However, the stress response indicators such as COR, NA, and GLU at T2 and T3 in the observation group were significantly lower than those in the control group. HR, MAP, SpO2, and other hemodynamic indexes were also significantly lower than those in the control group. These results show that sevoflurane is more helpful than propofol to reduce the stress response of surgery and anesthesia to the body and avoid excessive changes in hemodynamics. Considering the reasons may include the following aspects. First, the stress response caused by surgery, anesthesia, and other stimuli is mainly manifested as increased pituitary-adrenal cortex secretion and sympathetic nerve excitation, resulting in increased levels of NA, A, COR, increased heart rate, blood pressure, and blood sugar. The sevoflurane can inhibit the excitability of the parasympathetic nerve, and the analgesic effect of compound nerve block anesthesia can effectively reduce the stress response of the body. Second, sevoflurane combined nerve block anesthesia can effectively inhibit the production of catecholamines and can organize the opening of calcium ion channels and promote vasodilation. Sevoflurane can improve vascular endothelial function by acting on the vascular endothelium, promote the production of prostaglandins and nitric oxide and accelerate the relaxation of vascular endothelium. This can promote blood circulation and alleviate hemodynamic changes. In terms of cognitive function, sevoflurane also has significant advantages over propofol. In this study, the MMSE score of the observation group was significantly higher than that of the control group. The completion time of TMT was significantly shorter than that of the control group. These indicate that sevoflurane combined nerve block can significantly reduce the impact of surgical stress on the cognitive function of patients. This study also found that the incidence of adverse reactions in the observation group was significantly lower than that in the control group, indicating that sevoflurane combined nerve block can improve the safety of anesthesia and surgery. It is considered to be related to its mild stress response, stable hemodynamics, and quick postoperative recovery. The disadvantage of this study is that the effect of different sedation depths on the postoperative cognitive function of patients was not analyzed, and further research is needed in the later stage.

The article "Application Effect of Sevoflurane Combined with Nerve Block Anesthesia in Surgical Anesthesia in Patients with Uterine Fibroids" was published in 2022. Journal: Contrast Media Mol Imaging.

In conclusion, sevoflurane combined nerve block can significantly reduce the degree of stress response in patients undergoing laparoscopic myomectomy, maintain the relative stability of hemodynamics, and reduce the impact on postoperative cognitive function of patients. It improves the safety of anesthesia and surgery and is a relatively ideal way of anesthesia.

## Figures and Tables

**Table 1:** Comparison of general clinical data of two groups of patients.

Group	n	Age/year	Weight/kg	Disease duration/month	Fibroids size/cm
Observation	50	42.32 ± 5.01	58.73 ± 5.21	19.05 ± 0.87	5.04 ± 0.79
Comparison	50	42.35 ± 5.02	58.76 ± 5.25	19.08 ± 0.89	5.05 ± 0.80
*t*	—	0.03	0.03	0.17	0.06
*P*	—	>0.05	>0.05	>0.05	>0.05

**Table 2:** Comparison of surgery-related parameters between the two groups.

group	Number of patients	Anesthesia induction time	Operation time (min)	Blood loss (mL)
Observation	50	3.39 ± 0.62	131.45 ± 34.12	342.55 ± 51.22
Comparison	50	3.28 ± 0.55	124.98 ± 33.71	344.74 ± 43.65

**Table 3:** Comparison of stress response indicators between the two groups (*n* = 50).

Group	COR (ng/L)	A (ng/L)	NG (ng/L)	GLU (mmol/L)
Comparison				
T1	126.88 ± 14.95	187.45 ± 19.36	232.38 ± 21.03	4.94 ± 0.23
T2	211.39 ± 30.12^#^	238.65.39 ± 24.62^#^	342.49 ± 30.41^#^	6.90 ± 0.41^#^
T3	185.81 ± 20.43^#^	208.81 ± 21.59^#^	312.37 ± 20.94^#^	5.71 ± 0.28^#^
*F*	218.41	82.011	359.760	576.073
*P*	<0.01	<0.001	<0.001	<0.001

Observation				
T1	127.40 ± 16.84	187.30 ± 20.67	232.16 ± 17.66	4.94 ± 0.33
T2	134.49 ± 16.21^*∗*^^#^	201.59 ± 2.67^*∗*^^#^	255.91 ± 22.09^*∗*^^#^	5.25 ± 0.41^*∗*^^#^
T3	130.79 ± 14.71^*∗*^^#^	191.06 ± 16.69^*∗*^^#^	246.63 ± 23.49^*∗*^^#^	5.09 ± 0.23^*∗*^^#^
*F*	2.966	8.098	19.392	12.754
*P*	0.054	<0.001	<0.001	<0.001

^*∗*^Compared with the control group, *P* < 0.05; #compared with T1, *P* < 0.05.

**Table 4:** Comparison of hemodynamic indexes between the two groups (*n* = 50).

Group	HR (time/min)	MAP (mmHg)	SpO_2_ (%)
Comparison			
T1	81.31 ± 4.95	64.01 ± 6.27	97.57 ± 5.93
T2	90.01 ± 2.47^#^	78.93 ± 6.62^#^	108.34 ± 5.73^#^
T3	88.27 ± 2.81^#^	71.96 ± 4.29^#^	99.73 ± 5.33^#^
F	98.956	98.721	60.534
P	<0.01	<0.01	<0.01

Observation			
T1	81.27 ± 5.18	64.65 ± 5.90	98.24 ± 5.14
T2	84.69 ± 2.15^*∗*^^#^	70.61 ± 6.12^*∗*^^#^	103.96 ± 0.67^*∗*^^#^
T3	82.59 ± 2.71^*∗*^^#^	66.30 ± 5.19^*∗*^^#^	94.63 ± 5.49^*∗*^^#^
F	13.866	17.247	39.592
P	0.054	<0.001	<0.001

^*∗*^Compared with the control group, *P* < 0.05; #compared with T1, *P* < 0.05.

The article "Application Effect of Sevoflurane Combined with Nerve Block Anesthesia in Surgical Anesthesia in Patients with Uterine Fibroids" was published in 2022. Journal: Contrast Media Mol Imaging.

**Table 5:** Comparison of cognitive function between two groups (*n* = 50).

Group	MMSE (score)		TMT completion time (second)	
	1 day before surgery	1 day after surgery	1 day before surgery	1 day after surgery
Comparison	28.89 ± 0.43	25.28 ± 0.62^*∗*^	34.90 ± 1.70	39.36 ± 2.13^*∗*^
Observation	28.79 ± 0.39	27.97 ± 0.26	34.89 ± 1.80	35.20 ± 1.85
*t*	1.316	47.457	0.016	11.445
*p*	0.193	<0.001	0.987	<0.001

**Table 6:** Comparison of adverse reactions between the two groups (*n* = 50).

Group	Dizziness	Nausea and vomit	Lethargy	Restless	Total
Comparison	4 (6.67)	4 (6.67)	3 (5.00)	2 (3.33)	13 (21.67)
Observation	2 (3.33)	1 (1.67)	2 (3.33)	0 (0.00)	5 (8.33)
*X* ^2^	NA	NA	NA	NA	4.183
*P*	NA	NA	NA	NA	0.041

## Data Availability

The experimental data used to support the findings of this study are available from the corresponding author upon request.
